# Research on the Dominant and Implicit Integration Mechanism of Mental Health Education in Ideological and Political Education

**DOI:** 10.1155/2022/1356022

**Published:** 2022-04-13

**Authors:** Jing Xie

**Affiliations:** Ideological and Political Theory Teaching and Researching Department, Zhengzhou Railway Vocation and Technical College, Zhengzhou 451460, China

## Abstract

In order to improve the effectiveness, this article puts forward a research on the integration mechanism of explicit education and implicit education of psychological education in ideological and political education from the perspective of new media. Starting from the concept, characteristics, and types of new media, from the connotation, characteristics, theory, and practical significance of explicit education and recessive education, and from the perspective of new media, the integration mechanism of explicit education and recessive education in ideological and political education should be promoted. According to the integration principle of explicit education and implicit education in the new media perspective, this paper puts forward the integration strategy of explicit education and implicit education in the new media perspective. By using Marxist philosophy, instillation theory, and four learning theories, the paper uses the subjective sampling method to conduct a questionnaire survey on a university and puts forward some suggestions for the practical situation. The results show that the integration of explicit and implicit education into ideological and political education from the perspective of new media is effective and feasible, which can effectively improve the effectiveness of ideological and political education, promote the development of ideological and political education in university, and ensure the quality of ideological and political education in university.

## 1. Introduction

The new era of intelligent technology is gradually forming, and a variety of new network communication-based communication equipment in people's daily lives is constantly deepening [1]. Through different signs, it can be explained that people have been making progress. Under the guidance of deepening coverage project, network poverty alleviation project, and digital rural construction policy, the field of digital information has deepened [2, 3].

At present, traditional dominant education is not effective. For a long time, the ideological and political course, as the main position of explicit education in colleges and universities, has paid more attention to the knowledge and theory of classroom teaching, focusing on the one-way instillation of textbook knowledge step by step. The lack of communication between the teachers of ideological and political courses and the teachers of specialized courses and the lack of understanding of the characteristics of the majors studied by the students led to the lack of typical cases in the professional fields concerned by the students to enrich the teaching content of ideological and political courses, which ultimately greatly reduced the teaching effect of ideological and political courses and failed to effectively play the guiding function of the main channel of ideological and political education. Therefore, it has become a hot issue to study the integration mechanism of explicit education and implicit education. Since explicit education was put forward in 1990s, only some experts indirectly put forward the related concepts of explicit education. At first, people did not think it was an important way of education. Because different experts have different theoretical knowledge reserves and academic abilities, their understanding of explicit education has its own characteristics, which leads to the lack of unified definition of explicit education at present. Wang Ruisun's definition of explicit education is recognized by today's academic circles. He pointed out that explicit education of ideological and political education is an ideological and political education method organized and systematically carried out by various public places and means according to the instructions of leaders. In addition, some scholars also hold different views. They pointed out that explicit education is a scientific and systematic educational process, and it is an educational means actively and directly carried out among the public according to the wishes of organizations and leaders, combined with specific projects. In today's society, college students high activity and distinctive personalities. Due to its rich and humanized shape design and application concept, new media network is a platform widely accepted and applied by the majority of college students, with recessive education as the starting point, combined with explicit education, and news and current events and hot events as the basis [4]. This paper puts forward the integration strategy of explicit education and implicit education from the perspective of new media. Explicit education and implicit education, as two different aspects of ideological and political education in colleges and universities, can be vividly compared to hardware and software in ideological and political education in colleges and universities. Although explicit education and implicit education have their own characteristics, they also have their own shortcomings. In order to strengthen the role of ideological and political education, only by complementing the advantages and disadvantages of both can the best educational effect be achieved. Based on the analysis of the current new media background, this paper introduces new media technology into the ideological and political classroom in colleges and universities, strengthens the education of students, and achieves good ideological and political education effect.

## 2. Literature Review and Theoretical Research

### 2.1. New Media

#### 2.1.1. New Media Features

1. *Digitalization*. Digitalization is not only a means to realize new functions of new media but also different from traditional media in essence. For example, analog information is transformed into binary language by digital technology, and the “bit” form of separated information is transformed into 1 and 0 [5]. Different combinations of 1 and 0 series directly affect the decoding and reconstruction of separated information, thus presenting the original appearance. Digitization is a process in which all kinds of information are transformed into digital signals for transmission and are applied in comprehensive services [6], and then the receiver is used to restore its original transmission form, which can realize infinite recovery and avoid the damage of digital information. Digital technology belongs to the revolution of information processing [7]. Compared with the analog system of traditional media, new media can effectively use the unique advantages of the digital system.
2. *Interactivity*. The interactivity not only reflects the characteristics of human-computer interaction but also has the characteristics of machine. The characteristics mainly show that users can use computer-aided design to realize characteristics of using the machine to interact. The communication activities of new media belong to two-way informatization. Therefore, new media can not only transmit and receive information but also produce information.
3. *Unconventionality*. Unconventionality is one of the main characteristics of new media communication. Because “unconventionality” means negating or covering up the definition of “convention,” the premise of mastering unconventionality is to understand “convention.” Receive users using various media and channels according to users who initiate communications. Conventional communication is a form of one-way communication, which is characterized by uninterrupted and directional determination [8]. However, when reading the media information of printed matter, because of the limitation of space, it can only be read forward or backward. The process of implanting information into new media in the form of database is collocated and unconventional. In a structured way, the database is restored to a related or unrelated juxtaposition group, in which the propagation users directly affect the establishment of the juxtaposition group. That is, users can browse and consult digital information according to the relationship between digital information and different angles. The way to obtain information can be divergent or can be extended to all directions endlessly. The new media cannot use the method of controlling the amount, structure, and arrangement order of information, which limits the dissemination of users' information acceptance in time and space. Compared with traditional media, new media belong to a process that can realize and unify single line thinking and single sentence reduction to point structure and multiple sentences, so it is consistent with people's associative thinking mode.

#### 2.1.2. New Media Types

The forms of new media are very complex and numerous, and the communication modes formed by new media are also numerous. Among them, the most basic types of new media are mainly composed of the Internet, mobile terminal, digital TV, and other new media.

1. Internet new media: they refer to various forms of new media based on the Internet, mainly including web page, blog, network video, network broadcasting, and so on [9]. The Internet has evolved from a narrow and short group media form.
2. Mobile terminal new media: they refer to the use of mobile phones as the basis of receiving terminal communication form, which mainly includes mobile terminal SMS, mobile terminal newspaper, mobile terminal broadcast, etc. Because of its portability and mobility, the mobile terminal has greatly changed people's communication mode and information transmission mode, and its function is more and more powerful. Now mobile terminal telephone is not only a communication tool but also “fifth media,” second only to the traditional media.
3. Digital TV: users can also use digital TV to independently select TV programs and viewing time. Users can also use the digital TV receiver to interact with the broadcasting service terminal of the TV station to realize the service interface of online banking and online learning, so as to experience the one-to-one information service function.

### 2.2. Ideological and Political Education

It refers to the practice of the whole social group, which belongs to a common human behavior. It mainly adopts the relevant ideological, political, and moral standards and applies them to the relevant members with purpose, plan, and organization, so as to enable the relevant members to have the ideological and moral qualities needed by the specific society or class to a certain extent. To a certain extent, it defines the activities of the proletariat [10]. It belongs to different stages of common social activities, can help people further understand the objective necessity, and can also inherit and draw lessons from different classes in Chinese and foreign history, comparative criticism, and comparison of various useful experience.

### 2.3. Explicit Education

#### 2.3.1. Connotation of Explicit Education

The dominant education with authority and recognition is defined as “dominant education.” On this basis, education is offered in the form of teaching activities, theoretical lectures, and political situation reports. Specifically speaking, explicit education in education takes the classroom, which is theoretical, knowledgeable, and perceptive. At the same time, it is also a kind of teaching and social practice activity, with planning, goals, and direction.

The dominant education is also reflected in the development and application of the dominant curriculum. It refers to classroom teaching as the carrier, and the school has the ability to organize and systematically impart knowledge such as political theory, philosophy, moral theory, and so on. The teachers in university set the carrier as the classroom, set the teaching tools as a series of policies and regulations, philosophy, and ethics stipulated by the Ministry of Education, and teach the educated directly, visibly and consciously.

#### 2.3.2. Characteristics of Explicit Education

Education mainly puts explicit education in the first place. The dominant education has the following characteristics:

1. Clear educational purpose: the explicit education in education belongs to the implementation, mainly through the organization with plans and objectives. The implementer publicly explains the truth, viewpoint, and requirements to the educated object. At present, the educational object and the implementer have gradually accepted this traditional education.
2. Stabilizing the subject and object: educational subjectivity refers to the mutual clarification of their respective status and role. The main responsibility of implementers is to teach ideological and moral concepts, while that of objects is to accept these concepts, that is, the process of accepting the tasks of education implementers.
3. Open education mode: the dominant education must use various open means to show the educators' opinions and requirements in public places and then strive to use propaganda and direct explanation to achieve the unity of people's ideological purpose and expand the influence to a certain extent.
4. Integration of education content: the dominant education refers to the age of the educated, the ideological reality, and the needs of social situation [11]. Therefore, the logicality, scientificity, and integrity of the content have been effectively expanded. For example, the unity and comprehensiveness of ideological and political theory teaching, combined with the real-time nature of political conference discussion and reports, can realize the key role of education implementation and achieve the fundamental purpose of cultivating educational objects.
5. Simplifying educational behavior: explicit education refers to the use of unified organizational activities, so as to make the education information be quickly transmitted, so as to enhance the timeliness of information, make students understand the views and ideas of education implementers, and give timely feedback information.

#### 2.3.3. Practical Significance of Explicit Education

In university education, it cannot be completely realized, and the generation of moral consciousness must first be stimulated by a specific educational situation, from the outside to the inside gradually. In the early stage of moral development, individuals need to accumulate the basic knowledge of morality. Scholars in related fields have shown that only when the school imparts some value content to the education object, the education object can make some progress in the value field. However, if we cannot absorb all kinds of arguments and opinions effectively and firmly, the educational objects will have no good foundation to develop their value. Therefore, for a long time, dominant education has played a unique role in moral education.

The most active stage in life belongs to the state of university. In other words, it is the process from youth to adult, from simple development to maturity, from dependence to independence, from external environment to internal growth environment, and from individual to social group. Due to the influence of many factors such as western ideology and economic globalization, the ideology, consciousness, and ethics of college students are bound to be impacted [12].

We should use explicit education, so as to stimulate the potential awareness of the educational object, and seek truth from facts in the true sense, and actually touch real things, rather than the untouchable and illusory theoretical framework. On this basis, it is a practical task to cultivate qualified, sound, and high-quality contemporary college students with purpose and consciousness so as to improve their effect.

### 2.4. Recessive Education

#### 2.4.1. Connotation of Recessive Education

Recessive education is based on “recessive curriculum.” Hidden in the living environment and specific forms of activities around the education objects, they unconsciously accept the education professors to a certain extent and store their knowledge in the campus life other than theory curriculum education [13].

The form of recessive education does not directly affect the education object itself but often exists in the campus environment, humanistic environment, and various systems in the form of recessive education. This is a kind of educational model without representation. In the case of no specific educational goal and orientation, the use of behavior is totally unconscious and hidden, so that the educational object can learn, accept, and understand the theoretical concepts of consciousness and internalize the behavior norms of the educational object itself.

#### 2.4.2. Characteristics of Recessive Education

Implicit education refers to unconsciously grasp the education object consciousness and moral ethics, that is, recessive education can integrate the realm and emotion of education. For a contemporary college student, what really matters is the living environment around him. The main features are as follows:

1. In communication, educational individuals are not guided by their achievements but follow their own intentions under certain conditions. That is to say, they can decide each other's actions and decisions according to the principles stipulated by the common situation. For the implementers of education, whether it is in the social position or the knowledge reserves and experience accumulated by themselves, it has certain advantages compared with the educational object [14]. Often in the personality breakthrough, this superiority, the equal dialogue, pursues the education implementer and the education object itself. Education implementation has always been the main problem in the equal status relationship and plays a major role in the equal subject.
2. Diversified and extensive education carriers: the types of implicit education carriers in ideological and political education are complex and changeable, which widely exist in campus, humanities, and daily life environment. Recessive education carrier is mainly composed of material and culture. The material aspect refers to the existing environment. The cultural aspects include the history of the school, the school motto, and other practical activities. The system makes it more open, but this feedback does not mean that its application is arbitrary. These carriers must have two characteristics: the purpose of the educational implementer and the practical significance of the educational objects involved, so as to realize the diversity and wide education carrier in the real sense.
3. Implicit and infiltrating education content: because implicit education in ideological and political education belongs to non-representation education, education implementers always integrate implicit and infiltrating education content into education carrier. Also, it will be stored in the ideal environment created by the education implementer for the education object, so as to teach the education object imperceptibly to a certain extent, so as to achieve a real sense of psychological accumulation.

#### 2.4.3. Theoretical Basis of Implicit Education

British curriculum experts believe that “hidden curriculum” first appeared in Plato's time. As early as the turn of the century, American educational thinker and his students embodied the concept of “hidden curriculum.” The important embodiment of “indirect learning” is that the formation of emotional attitude directly affects future value. Further research on the learning process shows that holistic learning is mainly composed of direct learning, auxiliary learning, and indirect learning.

“Active learning” refers to the direct learning of things themselves, which belongs to the learning of directly acquired knowledge and skills. It also summarizes the ideals, attitudes, and moral habits to a certain extent, and the knowledge and skills are gradually mastered by students. “Auxiliary learning” refers to the continuous learning.

#### 2.4.4. Practical Significance of Implicit Education

On the basis of the emphasis of the recessive education, the infiltration mode of the recessive education should be strengthened, and the shortcomings of the hidden education should be compensated for by the indirect and covert features [15]. As the guide of advanced culture, college students can quickly grasp and directly affect their way of thinking. Information age provides new opportunities, quickly completes socialization, effectively uses modern information technology to consolidate status.

### 2.5. Research on Integration Strategy

Explicit education tends to pay more attention to pertinence and emphasis. It goes straight to the point and systematically imparts knowledge to people, which is conducive to the formation of educated knowledge system, so it has also become an educational method that educators use more. However, it is precisely because of its dominant characteristics that it will produce a sense of compulsion. This kind of educational method is too systematic and thorough, which often makes the educated feel bored and extremely tired, thus resulting in rejection. However, in the weak aspects of explicit education, implicit education is often promising. The biggest difference between implicit education and explicit education is that it hides the educational purpose and skillfully uses the psychological characteristics of the educated, so that the educated can unconsciously learn knowledge in the pleasant education process, thus achieving the expected educational effect. Because recessive education permeates and diffuses imperceptibly, it enters people's subconscious over time and makes the educational content deeply rooted in people's hearts. At the same time, implicit education also has its own shortcomings and deficiencies. Because of its lack of guidance, pertinence, and effectiveness, it cannot give an accurate and quick reply to some wrong thoughts and different puzzles, which will be very unfavorable to the formation of professional knowledge system and the strengthening of professional quality. In view of the above factors, in order to make the implicit education and explicit education produce excellent results, it is necessary to combine the advantages of implicit education and explicit education, which is also conducive to the moral education in colleges and universities.

#### 2.5.1. Integration Principle of Explicit Education and Implicit Education

The integration principles in the new media are as follows:

1. Latent: under normal circumstances, education exists mainly in the form of explicit education. The new media network is rich in information resources and knowledge and can provide sufficient survey data, which can be used as a reference for recessive education. Therefore, education implementers also need to research and develop, follow the principle of latency, in order to achieve the effective integration of the new media perspective, and achieve the effect of effective education for students.
2. Dynamic: due to the wide application information network, college students' access to information sources is increasing, and contemporary college students usually have their own specific needs and ideas. We need effective mutual assistance between education implementers and education objects. On this basis, to keep in touch with trends and trends, more long-term, more realistic treatment of the problem.
3. Diversification: because new media methods are applied by students, the educational communication path increases to a certain extent. The new media network is used to express the content of education network pictures or videos in the integration mechanism of explicit and implicit education of ideological and political education. Therefore, in education activities, education implementers need to effectively apply various forms of new media network and transmission path.
4. Selectivity: the network is a kind of fast and widely spread new media. If the amount of information is too large, students will receive more information and mental health. Combined with the reality of educational purpose, the new media network is constantly infiltrated.
5. Equivalence: students get ideological and moral education and have strong adaptability. At the same time, they are in a special psychological period. They pursue freedom, equality, and high independence and refuse passive learning. Therefore, combining explicit and implicit education in education, it is latent around students and provides a direct teaching place for implementation. Through non-face-to-face two-way interaction, let college students show their independent dominant position, pay attention to methods and means, and avoid students' negative feelings.

#### 2.5.2. Integration Strategy of Explicit Education and Implicit Education

Under the guidance of the goal of ideological and political education in colleges and universities, the unity of explicit education and implicit education is an organic whole which is composed of various links such as educational subject, educational content, educational object, educational form, and educational environment. At present, the international and domestic situation has undergone profound changes, and various ideologies and cultures in the ideological field have exchanged, blended, and confronted each other. Ideological and political education is facing many new tasks and challenges. In view of the problems existing in the current unification of explicit education and implicit education in China, the ideological and political education in colleges and universities can promote the unification of explicit education and implicit education from the following aspects, so as to strengthen the unification and integration of explicit education and implicit education and give full play to the role of ideological and political education in colleges and universities:

1. Change of educational concept: clearly understand the advantages of recessive education and truly understand education; if we can meet the above requirements, then we can effectively integrate explicit education and implicit education. China's people-oriented concept has not been put forward for a long time, but it can stand the test of the times. People-oriented concept is in line with the development trend of the times in today's international environment and era background, and it is also in line with the trend of the times. Generally speaking, we should adhere to the interests of the people and follow the wishes of the broad masses of people and the mainstream values. People-oriented concept requires us to pay attention to the way that educatees realize their self-worth and pay more attention to their needs for basic living materials. Educators in colleges and universities should have a correct understanding of the target and their orientation of the educated, understand their inner thoughts, take the improvement of the quality and all-round development of the educated as the direct work orientation, and finally turn the social needs into the intrinsic qualities of individuals, so as to promote the unity of explicit education and implicit education.
2. Education mode reform: combine the dominant education with recessive education and adopt the reformed education mode in the process of conveying ideas, so as to make the dominant education have higher persuasive ability and make the recessive education have higher efficiency. The dominant education is to create a good classroom atmosphere for teachers. When teachers carry out explicit education, they should integrate explicit education with recessive education according to their moral cultivation, so that students can learn to further display explicit education in class, and promote students' own personality qualities through the implementers of education. With the advent of today's Internet age, various software programs and platforms have been widely used as mass media. Accordingly, educators can use some videos and music to edify students in various forms. In addition, for some students who do not want to participate in the interaction in class, they can learn and communicate in real time through colorful pictures and videos on the Internet, so as to improve their learning enthusiasm, thus improving the effect of ideological and political education.
3. Development of educational resources: while students are learning and understanding the knowledge, they need to really identify the knowledge from both emotional and ideological aspects. In order to enhance students' self-confidence, in addition to making students master knowledge, we should integrate explicit and implicit education and show a more comprehensive education in the form of classroom platform, especially in the professional disciplines that need to infiltrate the concepts of morality and values. They can not only provide support for explicit education but also impart implicit education in a certain mode. We can provide students with educational edification and places and use campus activities to realize campus culture, so that to a certain extent, students have a high interest in participating in the activities, feel the activities in a real sense, and create a good and constantly improving cultural environment. The teaching content of the ideological and political education theory course is not only an important carrier of the course construction but also an important guarantee to enhance the affinity of the ideological and theoretical course and improve the teaching effect. At present, the renewal cycle of ideological and political textbooks is long, and the teaching content lags behind. Therefore, improving the freshness and flexibility of teaching content has become an important task for ideological and political talents in colleges and universities. First of all, the teachers of the ideological and political theory course should study, understand and apply realistically, and take various forms to enable the theory of socialism with Chinese characteristics in the new period to truly enter the classroom. Secondly, teachers of ideological and political courses should do everything from reality, pay attention to students' concerns, fully embody social hot and difficult issues in the teaching content through vivid and interesting teaching methods, and raise students' own meager theoretical knowledge to a new height. Thirdly, teachers should constantly improve teaching methods, make full use of comparative education methods through analyzing the national and world situation, compare socialist society with Chinese characteristics with capitalist society, answer and solve social hot issues, and cultivate the historical mission and national identity of talents in the new era through the combination of explicit and implicit education.
4. Educational activities: we should combine explicit education with implicit education in education to improve the efficiency of knowledge transfer. One is to carry out activities, use science and technology to enrich educational resources, obtain unlimited educational knowledge anytime and anywhere, recessive educational atmosphere, and provide effective places. The second is to carry out online activities based on the new media network and help schools, education implementers, and even education objects to better develop ideological and political education. Teachers engaged in ideological and political education in colleges and universities should correctly recognize the important role of integrating theory with practice, an important essence of Marxist thought, and carry out ideological and political teaching on this basis. Political teachers should not only pay attention to teaching students the knowledge in books but also arrange students to carry out social practice activities. By visiting the enterprise, let them understand how the theoretical knowledge learned in books is applied in practice. Through the visit to the Red Revolutionary Base, they can learn the fearless spirit of revolutionary martyrs' hard work in the past arduous environment and their dedication to the motherland. In class, teachers should impart theoretical knowledge to students according to the content of teaching materials. Outside the classroom, teachers should lead students to organize social practice tasks of various natures, divide students into different groups to discuss their learning experiences, and make special PPT through division of labor, which will be displayed and exchanged in turn in the classroom, so as to strengthen students' theoretical knowledge.

## 3. Empirical Analysis

### 3.1. Data Sources

A polytechnic university is taken as an example. In this paper, the integration mechanism of explicit education and implicit education is applied to this university education. Colleges and universities should strengthen the research and utilization of new media means for students such as Tik Tok and Volg, establish campus all-media centers, make good use of school newspapers, official websites, WeChat, microblog, and official Tik Tok, and actively build all-media platforms to guide new media to play an active role in ideological and political education of college students. The respondents are all college students. The questionnaire is conducted by subjective sampling. A total of 1048 questionnaires were issued and 1025 were recovered. After eliminating the invalid questionnaires, 1012 valid questionnaires were obtained. The effective recovery was 96.5%. This study mainly uses SPSS13.0 statistical analysis and processing data, using univariate description statistical analysis of relevant data.

### 3.2. Sample Characteristics

In this paper, EViews and other statistical software are used to establish the database and make statistics on the effective samples. The results are shown in Table 1.

According to the data in Table 1, there were 586 male college students, accounting for 57.9%, 426 female college students, accounting for 42.1%, and 267 freshmen, accounting for 26.4%. There were 259 sophomores, accounting for 25.6%. There were 247 junior students, accounting for 24.4%. There were 239 senior students, accounting for 23.6%.

### 3.3. Integration of Explicit and Implicit Education

This paper analyzes the current situation of the integration of explicit and implicit education, so as to make better use of new media and make students affected.

1. The information sources of college students are given in Table 2.
2. It can be seen from the data in Table 2 that 784 college students obtained information from the Internet, accounting for 77.5%; 85 college students got information from TV, accounting for 8.4%; 58 college students got information from newspapers, accounting for 5.7%; and 49 students got information from the classroom, accounting for 4.8%. There are 36 college students who get information from books, accounting for 3.6%. From this, we can see that the information is mainly through the network, and the proportion is more than 70%.
3. The Internet time of college students is given in Table 3.
4. According to the data in Table 3, 354 college students spent less than 2 hours online, accounting for 34.9%; 487 college students spent 2–5 hours online, accounting for 48.1%; 83 college students spent 5–8 hours online, accounting for 8.2%; 69 college students spent more than 8 hours online, accounting for 6.8%; and 19 college students spent 0 hours online, accounting for 1.8%. It can be seen that 98.2% of college students have access to the Internet, indicating the popularity of new media networks among college students. Among these students, more than half of them spent 2–5 hours on the Internet, which shows that the Internet time accounts for a large proportion of their study time.
5. The contents of college students' online browsing are given in Table 4.
6. As can be seen from the data in Table 4, there were 247 college students browsing the Internet for chat, accounting for 24.4%. There were 135 college students browsing microblog online, accounting for 13.3%. There were 158 college students browsing games online, accounting for 15.6%, and 239 college students read news online, accounting for 23.6%. There were 114 college students browsing online for shopping, accounting for 11.3%. There were 119 college students who browsed the Internet to watch plays, accounting for 11.8%.
7. The influence of college students on the Internet is given in Table 5.
8. It can be seen from the data in Table 5 that 241 college students were always influenced by the Internet, accounting for 23.8%, and 726 college students were occasionally influenced by the Internet, accounting for 71.7%. There are 45 college students who have no influence on the Internet, accounting for 4.4%. It can be seen that 95.6% of college students will be affected by the Internet compared with those who will never be affected by the Internet. Therefore, it is feasible to integrate explicit and implicit education. Practice has proved that the ideological and political explicit education can make full use of new media means and make overall use of all kinds of resources, Change the traditional teaching mode of teachers' single words, full time, and students' lack of initiative and constantly meet the needs and expectations of students' growth and development.

### 3.4. Attribution Analysis of the Integration of Explicit and Implicit Education

From the perspective of new media, the main conditions are diversified network content and presentation forms. However, the current perspective is the lack of this content, resulting in monotonous network content. In addition, the content presentation is mostly text-based, lacking other types. In today's information age, education implementers need to use a large number of new media images to enable students to accept education in the integration mechanism. The contents and forms are given in Figures 1 and 2.

As can be seen from Figure 2, education covers more forms. Students' requirements for educational methods. Therefore, from the perspective of new media, it is also necessary to innovate the forms of reports, establish the integration mechanism of explicit education and implicit education, strengthen educational links and interactive exchanges, and promote university education.

## 4. Conclusion and Discussion

This paper takes the students of a university of science and technology as the research object and makes an empirical analysis of the integration mechanism of explicit and implicit education in ideological and political education from the perspective of new media. This paper has the following findings and reflections:

1. By analyzing the content of the questionnaire, it is concluded that the integration effect of explicit and implicit education is better. The new media network has a high popularity among college students, and the online time accounts for a large proportion of their study time. College students also pay attention to the national current affairs news to a certain extent. From the perspective of new media, the integration of explicit and implicit education in ideological and political education is feasible.
2. Through attribution analysis of the current situation of integration mechanism, it is concluded that education should start from many aspects to improve the effectiveness. From the angle of view, it also innovates its cover form, establishes integration mechanism, and strengthens education contact and interactive communication.
3. The paper found that the integration of explicit education and implicit education under new media can promote ideological and political education to a certain extent. In the future research, we should also consider strengthening ideological and political education as the starting point, integrate new media technology into education and teaching concepts, teaching methods, and professional teaching contents, and build a comprehensive ideological and political education system.

## Figures and Tables

**Figure 1:** Contents of ideological and political education.

**Figure 2:** The forms of ideological and political education.

**Table 1:** Basic characteristics of survey samples.

Sample characteristics (*N* = 1012)		Number (person)	Proportion (%)
*Gender*	Male	586	57.9
	Female	426	42.1

*Grade*	Freshman	267	26.4
	Sophomore	259	25.6
	Junior	247	24.4
	Senior	239	23.6

**Table 2:** Sources of college students' information.

Source of acquisition (*N* = 1012)	Number (person)	Proportion (%)
Network	784	77.5
Television	85	8.4
Newspaper	58	5.7
Classroom	49	4.8
Book	36	3.6

**Table 3:** Internet time of college students.

Online time (*N* = 1012)	Number (person)	Proportion (%)
<2 hours	354	34.9
2–5 hours	487	48.1
5–8 hours	83	8.2
More than 8 hours	69	6.8
0 hours	19	1.8

**Table 4:** Internet browsing contents of college students.

Browsing content (*N* = 1012)	Number (person)	Proportion (%)
Chat	247	24.4
Microblog	135	13.3
Game	158	15.6
Journalism	239	23.6
Shopping	114	11.3
Watch a play	119	11.8

**Table 5:** The influence of the internet on college students.

Impact (*N* = 1012)	Number (person)	Proportion (%)
Always	241	23.8
Occasionally	726	71.7
Never	45	4.4

## Data Availability

The datasets used and/or analyzed during the current study are available from the corresponding author on reasonable request.
